The article "Effectiveness of Laparoscopic Cholecystectomy in Patients with Gallbladder Stones with Chronic Cholecystitis" was retracted in 2023. Reasons: unreliable results or conclusions; concerns about the data; concerns about the peer review; concerns about the citations.

# Effectiveness of Laparoscopic Cholecystectomy in Patients with Gallbladder Stones with Chronic Cholecystitis

**DOI:** 10.1155/2022/1434410

**Published:** 2022-08-05

**Authors:** Leiping Rao, Guoqing Zhou, Yongzhong Gao, Yongchuan Huang, Hongwei He, Qiyun Gu

**Affiliations:** Department of Hepatobiliary and Pancreatic Surgery, Jinshan Branch of Shanghai the Sixth People's Hospital, Shanghai 201599, China

## Abstract

**Objective:**

To assess the effectiveness of laparoscopic cholecystectomy in patients with gallbladder stones and chronic cholecystitis.

**Methods:**

From July 2018 to January 2020, 90 patients with gallbladder stones and chronic cholecystitis assessed for eligibility were recruited and concurrently assigned (1 : 1) to receive either small-incision cholecystectomy (observation group) or laparoscopic cholecystectomy (experimental group). Outcome measures included operation time, intraoperative bleeding volume, postoperative hospital stay, c-reactive protein (CRP), interleukin (IL)-6, tumor necrosis factor-*α* (TNF-*α*), gastrin (GAS), vasoactive intestinal peptide (VIP), motilin (MOT), and adverse events.

**Results:**

Patients given laparoscopic cholecystectomy showed lower levels of operation-related indices versus those receiving small-incision cholecystectomy (*P* < 0.05). Laparoscopic cholecystectomy resulted in lower postoperative levels of CRP, IL-6, and TNF-*α* in the patients versus small-incision cholecystectomy (*P* < 0.05). Patients receiving laparoscopic cholecystectomy showed better GAS, VIP, and MOT levels than those receiving small-incision cholecystectomy (*P* < 0.05). The eligible patients after laparoscopic cholecystectomy had a significantly lower incidence of adverse events versus those after small-incision cholecystectomy (*P* < 0.05).

**Conclusion:**

Laparoscopic cholecystectomy effectively shortens the operative time and length of hospital stay in patients with gallbladder stones and chronic cholecystitis, reduces intraoperative bleeding, attenuates the inflammatory response, and enhances the gastrointestinal function, with less surgical trauma and high safety. Clinical trials are, however, required prior to promotion.

## 1. Introduction

Gallbladder stones are mainly formed by bile compounds in the gallbladder with high prevalence and multiple complications. Chronic cholecystitis is a common complication of gallbladder stones [1] and is attributed to tissue fibrosis elicited by repeated irritation of the mucosal epithelial tissue of the gallbladder by bile. Delayed medical management may lead to gallbladder perforation and acute peritonitis [2]. Cholecystectomy is the most common procedure in hepatobiliary surgery. With the development of medical technology, minimally invasive surgery has captured more clinical attention [3], which has resulted in the substitution of traditional open cholecystectomy by small-incision cholecystectomy and laparoscopic cholecystectomy [4], both of which are considered safe and classical procedures [5]. However, it has been reported that small-incision cholecystectomy is associated with larger trauma versus laparoscopic cholecystectomy [6], which compromises patient prognosis. In addition, laparoscopic cholecystectomy is less prone to injuries to the gastrointestinal wall, greater omentum, and peritoneum during operation [7], which avoids intraoperative hemorrhage and suggests a higher safety profile versus small-incision cholecystectomy [8]. Accordingly, 90 patients with gallbladder stones and chronic cholecystitis from July 2018 to January 2020 were recruited to investigate the efficacy of small-incision cholecystectomy or laparoscopic cholecystectomy, thereby assessing the effectiveness of laparoscopic cholecystectomy in patients with gallbladder stones and chronic cholecystitis.

## 2. Materials and Methods

### 2.1. Baseline Data

From July 2018 to January 2020, 90 patients with gallbladder stones and chronic cholecystitis were recruited and assigned to two groups via the random number table method using the SPSS 23.0 software. Undersigned informed consent was obtained from the patients prior to enrollment. The study protocol was approved by the hospital ethics committee (ethical approval number JFJ20180728), and all processes complied with the Declaration of Helsinki's ethical guidelines for clinical research.

### 2.2. Inclusion and Exclusion Criteria

Inclusion criteria: patients who met the diagnostic criteria of the Consensus Opinion on Internal Medicine for Chronic Cholecystitis and Gallbladder Stones in China (2018) were included.

Exclusion criteria: patients with hepatocellular carcinoma or cirrhosis, with contraindications to surgery, with heart, liver, kidney, and other vital organ dysfunction, with a history of severe allergies, with severe hematological diseases, malignant tumors, or endocrine system diseases, in lactation or pregnancy, or with severe mental disorders were excluded.

### 2.3. Surgical Methods

The patients were given anesthesia in the supine position after routine disinfection, draping, and tracheal intubation.

The patients in the observation group were given small-incision cholecystectomy. A 5 cm incision was made below the right costal margin, the abdominal wall was incised layer by layer, and the tissue was separated to expose the surgical field. The gallbladder artery and cystic duct were dissected and ligated, followed by resection of the gallbladder, hemostasis, layer-by-layer suturing, and routine postoperative drainage.

The patients in the experimental group underwent laparoscopic cholecystectomy. An incision was made at the inferior border of the umbilicus, and a Veress needle was inserted, followed by the establishment of a CO_2_ pneumoperitoneum and the placement of a laparoscope to inspect the gallbladder, common bile duct, and Calot's triangle. Under endoscopy, the needle was inserted in the anterior axillary line, around the umbilicus, and 2 cm below the right side of the xiphoid process, followed by the dissection of Calot's triangle and the separation of the gallbladder ducts and vessels using an electrocoagulation hook. The gallbladder was resected and removed following a subxiphoid puncture, followed by the release of the pneumoperitoneum, hemostasis, layer-by-layer suturing, and routine postoperative placement of a drainage tube.

### 2.4. Outcome Measures

1. Operation indices: the operative time, intraoperative bleeding volume, and postoperative length of hospital stay were recorded
2. Serum inflammatory factor indices and serum gastrointestinal hormone levels: before and after surgery, 5 ml of fasting venous blood was collected from the patients in both groups and centrifuged at 3000 r/min for 10 min to obtain serum. The levels of c-reactive protein (CRP), interleukin (IL)-6, tumor necrosis factor-*α* (TNF-*α*), gastrin (GAS), vasoactive intestinal peptide (VIP), and motilin (MOT) of patients were determined by ELISA. The kits were provided by Beijing Wantai Biological Pharmaceutical Co., and were operated in strict accordance with the kit instructions.
3. Adverse events: postoperative adverse events including incisional infection, bile leak, pneumonia, and bleeding were recorded

### 2.5. Statistical Analysis

SPSS 22.0 was used for data analyses. The measurement data were expressed as ($\bar{x}$ ± *s*) and processed using the *t*-test. The count data were expressed as the number of cases (rate) and analyzed using the chi-square test. Differences were considered statistically significant at *P* < 0.05.

## 3. Results

### 3.1. Baseline Data

In the observation group, there were 24 males and 21 females, aged 37–61 (46.52 ± 5.37) years, with a duration of disease of 1–7 (4.21 ± 1.54) years, a BMI of 22–29 (25.12 ± 1.72) kg/m^2^, and a gallstone diameter of 2.5–16.9 (10.21 ± 2.32) mm. In the experimental group, there were 25 males and 20 females, aged 38–60 (46.63 ± 5.35) years, with a duration of disease of 1–8 (4.45 ± 1.50) years, a BMI of 22–29 (25.21 ± 1.68) kg/m^2^, and a gallstone diameter of 2.5–16.7 (10.14 ± 2.28) mm (Table 1).

### 3.2. Operation Indices

Patients given laparoscopic cholecystectomy showed lower levels of operation-related indices versus those receiving small-incision cholecystectomy (*P* < 0.05) (Table 2).

### 3.3. Inflammatory Factor Levels

Laparoscopic cholecystectomy resulted in lower postoperative levels of CRP, IL-6, and TNF-*α* in patients versus small-incision cholecystectomy (*P* < 0.05) (Table 3).

### 3.4. Serum Gastrointestinal Hormone Levels

Patients receiving laparoscopic cholecystectomy showed better outcomes of GAS, VIP, and MOT levels than those receiving small-incision cholecystectomy (*P* < 0.05) (Table 4).

### 3.5. Adverse Events

The eligible patients after laparoscopic cholecystectomy had a significantly lower incidence of adverse events versus those after small-incision cholecystectomy (*P* < 0.05) (Table 5).

## 4. Discussion

The development of gallbladder stones with chronic cholecystitis in patients is usually associated with excessive accumulation of bile salts and high cholesterol [9]. An imbalance in the ratio of cholesterol content and bile acids may lead to excessive storage of cholesterol in the bile, resulting in bacterial infection and precipitation [10] and gallbladder stones with chronic cholecystitis. Symptoms of gallbladder stones with chronic cholecystitis include abdominal distension and belching, and the lack of timely treatment may deteriorate the condition [11] and result in complications such as gallbladder effusion, obstructive jaundice, and porcelain-like gallbladder, seriously compromising the quality of life of patients [12]. Previously, open cholecystectomy is a common clinical treatment for gallbladder stones with chronic cholecystitis, but its efficiency is compromised by a large surgical trauma, long operative time, excessive bleeding volume, and a high risk of incisional infection. Small-incision cholecystectomy, modified from traditional open surgery, reduces the surgical incision and the risk of infection [13] but is limited by its narrow intraoperative field. Clinical research has confirmed that laparoscopic cholecystectomy provides the larger surgical field and contributes to the rapid removal of the lesion, significantly shortens the operative time and postoperative hospital stay, and promotes postoperative recovery [14]. A study by Alexander et al. suggested that laparoscopic cholecystectomy is less prone to medically induced injury to the gastrointestinal wall, greater omentum, and peritoneum during the operation and avoids intraoperative hemorrhage [15], and the closure of the gallbladder artery using an absorbable clip during the procedure significantly reduces intraoperative bleeding volume [16].

In the present study, patients given laparoscopic cholecystectomy showed lower levels of operation-related indices versus those receiving small-incision cholecystectomy, indicating that laparoscopic cholecystectomy effectively shortened the operative time and postoperative hospital days and reduced the intraoperative bleeding volume in patients. Moreover, the eligible patients herein after laparoscopic cholecystectomy had a significantly lower incidence of adverse events versus after small-incision cholecystectomy, suggesting a high safety profile of laparoscopic cholecystectomy, as laparoscopic cholecystectomy minimizes the exposure of the patient's internal organs and effectively avoids bacterial invasion [17]. In contrast to experimental results, research has shown that laparoscopic cholecystectomy is not suitable for complicated cases, such as severe adhesions in and around the gallbladder or concomitant common bile duct stones, and forced separation may lead to acute bleeding and metastasis [18]. The reason for the discrepancy may be that the continuous development of equipment and technology may affect the results and that there are differences in the constitution of the patients and the operations of the doctors in different regions. A relevant study showed that surgery is associated with impaired hepatobiliary function in patients with gallbladder stones and chronic cholecystitis, leading to inflammatory responses [18]. Reitano et al. stated that serum levels of inflammatory factors CRP, IL-6, and TNF-*α* directly reflect the degree of damage to surgical tissues, and patients with gallbladder stones and chronic cholecystitis showed abnormally elevated levels of serum CRP, IL-6, and TNF-*α* [19]. Here, laparoscopic cholecystectomy resulted in lower postoperative levels of CRP, IL-6, and TNF-*α* in patients versus small-incision cholecystectomy, suggesting that laparoscopic cholecystectomy is more effective in alleviating the inflammatory response in patients with gallbladder stones and chronic cholecystitis versus small-incision cholecystectomy, which may be attributable to the mild damage to hepatobiliary function and the low surgical trauma during laparoscopic cholecystectomy [20]. In addition, relevant studies have found varying degrees of gastrointestinal impairment in patients with gallbladder stones and chronic cholecystitis. In the present study, laparoscopic cholecystectomy resulted in better outcomes of GAS, VIP, and MOT levels, suggesting a more significant enrichment of serum gastrointestinal hormone levels benefits in patients with gallbladder stones and chronic cholecystitis by laparoscopic cholecystectomy versus small-incision cholecystectomy, probably because laparoscopic cholecystectomy is performed in a closed abdominal cavity, which effectively prevents prolonged exposure of the patient's gastrointestinal tract and promotes postoperative out-of-bed activities and postoperative recovery of the patient's gastrointestinal function [21].

IL-6 is a multifunctional glycoprotein consisting of 184 amino acids that can reflect the state of the body's response to inflammation and infection and is highly expressed in the bile and serum of patients with chronic cholecystitis [22, 23]. The local inflammatory response of the gallbladder is an important basis for the development of cholecystitis, and effective control of inflammation contributes significantly to the treatment of cholecystitis. The positive expression of EGFR in gallbladder cancer tissues was 70.7% and 85.7% in gallbladder atypical hyperplasia tissues, while there was no positive expression in normal gallbladder tissues, speculating that there may be a close relationship between EGFR and the development of chronic cholecystitis and gallbladder cancer [24]. Although this study provides certain ideas for treatment, a combination of Chinese and Western medicine may have better efficacy considering the existing drawbacks.

In TCM, acute cholecystitis is considered as internal heat, with the main location of the disease in the liver and gallbladder [25]. Acute calculous cholecystitis is classified as “biliary distension” and “jaundice,” which is mainly caused by internal dampness and heat due to liver qi stagnation, resulting in an imbalance of biliary function and qi flow and the formation of stones [26]. Currently, the preferred treatment is cholecystectomy, with the advantages of less trauma and bleeding, but the postoperative recovery is lengthy and painful, and there is a high risk of postoperative recurrence [27]. Chinese herbal medicine for the treatment of acute cholecystitis includes Longdan Xiegan decoction, Dachaihu decoction, Dachengqi decoction, and Jinling Sini powder, among which Dachaihu decoction is mainly adopted as the main formula with proper adjustment of the dosage of partial herbs, and the decoction is effective for elderly patients with acute cholecystitis of the damp-heat in the liver and gallbladder [28]. For painful symptoms of acute cholecystitis, acupuncture is usually performed at the Yanglingquan point to obtain significant pain relief [29].

## 5. Conclusion

Laparoscopic cholecystectomy effectively shortens the operative time and length of hospital stay in patients with gallbladder stones and chronic cholecystitis, reduces intraoperative bleeding, attenuates the inflammatory response, and enhances the gastrointestinal function with less surgical trauma and high safety. Clinical trials are, however, required prior to promotion.

## Figures and Tables

**Table 1:** Comparison of baseline data (*n* (%)).

	Observation group (*n* = 45)	Experimental group (*n* = 45)	*t* or *x*^2^	*P* value
Gender			0.045	0.832
Male	24	25		
Female	21	20		
Mean age (year)	46.52 ± 5.37	46.63 ± 5.35	−0.097	0.923
Mean duration of disease	4.21 ± 1.54	4.45 ± 1.50	−0.749	0.456
BMI (kg/m^2^)	25.12 ± 1.72	25.21 ± 1.68	−0.251	0.802
Gallstone diameter (mm)	10.21 ± 2.32	10.14 ± 2.28	0.144	0.886

**Table 2:** Comparison of operation-related indices ($\bar{x}$ ± *s*).

Groups	*n*	Operative time (min)	Intraoperative bleeding volume (mL)	Postoperative hospital stay (d)
Observation group	45	95.42 ± 7.81	123.14 ± 22.64	7.38 ± 2.57
Experimental group	45	61.24 ± 6.28	43.58 ± 14.50	5.39 ± 1.41
*T* value	—	22.879	19.851	4.554
*P* value	—	<0.001	<0.001	<0.001

**Table 3:** Comparison of inflammatory factor levels ($\bar{x}$ ± *s*).

Groups	*n*	CRP (ng/L)		IL-6 (ng/L)		TNF-*α* (*μ*g/L)	
		Preoperative	Postoperative	Preoperative	Postoperative	Preoperative	Postoperative
Observation group	45	42.17 ± 8.26	35.61 ± 7.60	55.32 ± 6.38	47.82 ± 6.38	7.53 ± 1.81	4.75 ± 0.92
Experimental group	45	42.24 ± 8.32	28.46 ± 8.11	55.41 ± 6.29	42.41 ± 5.72	7.47 ± 1.74	1.98 ± 0.77
*T* value	—	−0.04	4.315	−0.067	4.235	0.16	15.489
*P* value	—	0.968	<0.001	0.947	<0.001	0.873	<0.001

**Table 4:** Comparison of serum gastrointestinal hormone levels ($\bar{x}$ ± *s*).

Groups	*n*	GAS (ng/L)		VIP (ng/L)		MOT (pg/mL)	
		Preoperative	Postoperative	Preoperative	Postoperative	Preoperative	Postoperative
Observation group	45	93.54 ± 7.47	111.42 ± 10.35	24.76 ± 6.59	22.18 ± 5.26	141.65 ± 53.79	198.58 ± 43.29
Experimental group	45	93.48 ± 7.32	130.52 ± 13.21	24.89 ± 6.44	18.31 ± 3.68	141.53 ± 53.87	240.30 ± 38.94
*t*	—	0.038	−7.635	−0.095	4.044	0.011	−4.806
*P*	—	0.97	<0.001	0.925	<0.001	0.991	<0.001

**Table 5:** Comparison of adverse events (*n* (%)).

	Observation group (*n* = 45)	Experimental group (*n* = 45)	*x* ^2^	*P*
Incisional infection	2	1		
Bile leak	1	0		
Pneumonia	1	0		
Hemorrhage	4	1		
Incidence (%)	8 (18%)	2 (4%)	10.01	0.002
